# Prevalence of *algD*, *pslD*, *pelF*, *Ppgl*, and *PAPI-1* Genes Involved in Biofilm Formation in Clinical *Pseudomonas aeruginosa* Strains

**DOI:** 10.1155/2022/1716087

**Published:** 2022-05-24

**Authors:** Hakime Rajabi, Himen Salimizand, Mazaher Khodabandehloo, Amirhossein Fayyazi, Rashid Ramazanzadeh

**Affiliations:** ^1^Cellular and Molecular Research Center, Kurdistan University of Medical Sciences, Sanandaj, Iran; ^2^Department of Microbiology, School of Medicine, Kurdistan University of Medical Sciences, Sanandaj, Iran; ^3^Department of Microbiology, School of Medicine, Shahid Beheshti University of Medical Sciences, Tehran, Iran; ^4^Department of Microbiology, School of Medicine, Ardabil University of Medical Sciences, Ardabil, Iran

## Abstract

**Introduction:**

Biofilm formation is one of the main virulence factors in *Pseudomonas aeruginosa* infections. This study is aimed at investigating the presence of genes involved in biofilm formation in clinical *P. aeruginosa* isolates. *Material and Methods*. A cross-sectional study was conducted on 112 *P. aeruginosa* isolates. The biofilm formation assay was performed on all isolates. Antimicrobial resistance was determined by the disk diffusion method, and the presence of genes was detected by polymerase chain reaction. Isolates were typed with Rep-PCR.

**Results:**

The results of biofilm formation demonstrated that 85 strains (75.9%) were biofilm producers, and 27 strains (24.1%) were nonproducer isolates. Antibiotic susceptibility pattern in biofilm-positive and biofilm-negative isolates obtained from hospitalized patients showed a high rate of antibiotic resistance to amoxicillin with 95.7% and 92.3%, respectively. Based on PCR amplification results, the frequency of genes involved in biofilm formation among all isolates was as follows: *algD* (78.6%), *pelF* (70.5%), *pslD* (36.6%), *Ppgl* (0%), and *PAPI-1* (77.6%). Rep-PCR typing demonstrated that 112 *P. aeruginosa* isolates were classified into 57 types according to 70% cut-off. The predominant type was A which contained 15 isolates. Moreover, 7 isolates were clustered in genotype B, followed by C type (6), D (4), E (4), F (4), G (4), H (3), I (3), J (3 isolates), and 12 genotypes, each containing two isolates. Also, 35 isolates were distributed in scattered patterns and showed single types.

**Conclusion:**

Study results showed significant association between biofilm formation and resistance to antibiotics such as ceftazidime and meropenem. Analysis of Rep-PCR patterns indicated that the evaluated isolates were heterogeneous, relatively.

## 1. Introduction

*Pseudomonas aeruginosa* is a nonfermenting aerobic gram-negative and rod-shaped bacterium, which is reported to be omnipresent in the natural environment, animals, and humans [1]. *P. aeruginosa* is an important opportunistic pathogen that causes severe infections in immunocompromised patients and patients with neutropenia, cystic fibrosis, or severe burns [1]. Also, it is a major cause of healthcare-associated infections, routinely in intensive-care units [2]. Patients with cystic fibrosis (CF) are especially susceptible to chronic *P. aeruginosa* infections that can be leading to decreased lung function [3].

Biofilm causes bacteria to become resistant to a variety of antibiotics and disinfectants, which can lead to multidrug-resistant (MDR) strains [4]. Prevalence of MDR *P. aeruginosa* infections is the main concern of *P. aeruginosa* infection control, and treatment is more difficult [5]. The typical definition of a biofilm includes a community of bacteria adhered to a surface encased in a self-produced matrix [6]. *P. aeruginosa* develops these biofilms in the environment, on catheters, and in living tissues [7]. The biofilm structure is composed of the exopolysaccharides alginate, *Pel*, and *Psl* [8].

Alginate is a polymer including *α*-L-guluronic acid and *β*-D-mannuronic acid and has a significant role in the protection and structural stability of biofilm [9]. Most of the alginate-producing genes are located in a large operon [9]. The first gene in this operon is *algD*, which is necessary for alginate production, and its expression is completely controlled [10]. Another polysaccharide is *Psl*, which is composed of a repeating pentasaccharide, including L-rhamnose, D-glucose, and D-mannose [9]. *Psl* is essential at the beginning of biofilm formation and stability of biofilm structure [9]. The third polysaccharide is *Pel*, which is present in the biofilm of *P. aeruginosa* and is glucose-rich [11]. Furthermore, many surface proteins are involved in the formation of *P. aeruginosa* biofilm [11].

Another agent that has been shown to play a role in biofilm formation through structural and functional studies is the PpgL protein (periplasmic protein gluconolactonase—a protein that plays the role of gluconolactonase in the bacterial periplasmic region) [12]. This protein is encoded by the PA4204 gene, which plays a vital role in normal bacterial growth and biofilm formation [12]. PpgL protein is located in the periplasm and has gluconolactonase activity, which is why this protein is named [12]. This protein is predicted to belong to the propeller fold-*β* family, which has a normally compact structure with different cellular functions [12].

*P. aeruginosa* has two pathogenicity islands including PAPI-1 (108 kb) and PAPI-2 (11 kb) [13]. The PAPI-1 and PAPI-2 genes are located next to the lysine tRNA gene. PAPI-1 plays an important role in pathogenesis and the spread of disease, and many infections in the cell are due to the presence of this gene, so it can increase chronic infection in cystic fibrosis patients [13–15]. PAPI-1 encodes several regulatory genes, including PvrR, a two-component response regulator involved in antibiotic resistance and biofilm formation [16].

Various molecular methods, such as repetitive extragenic palindromic PCR (Rep-PCR), pulse-field gel electrophoresis (PFGE), and ribotyping have been used to evaluate the genotypic diversity of several bacterial species [17]. Recent studies have shown that Rep-PCR is a reliable and fast tool for differentiating and typing gram-negative bacteria such as *P. aeruginosa* [17].

Considering the importance of biofilm formation in pathogenicity and antibiotic resistance on the one hand and the important role of *algD*, *pslD*, *pelF*, *Ppgl*, and *PAPI-1* genes in biofilm formation, on the other hand, this study is aimed at investigating biofilm formation and the prevalence of these genes in *P. aeruginosa* strains. The clonal relationship for finding the origin of infection of the isolates was also evaluated with Rep-PCR.

## 2. Materials and Methods

### 2.1. Bacterial Collection

A cross-sectional study was conducted on 112 *P. aeruginosa* isolates between January 2020 and March 2021 in Sanandaj, Iran. Bacterial strains retrieved from the study of Ahmadi et al. (IR.MUK.REC.1397.269) are isolated from patients with *P. aeruginosa* infections of five cities (Zanjan: 40, Sanandaj: 31, Hamadan: 15, Zahedan: 14, and Mashhad: 12 isolates) of Iran. This study was evaluated and approved by the Ethics Committee of Kurdistan University of Medical Sciences (IR.MUK.REC.1398.259).

### 2.2. Antimicrobial Susceptibility Testing

The antibiotic susceptibility pattern was determined based on the disk diffusion method on Mueller–Hinton agar (Himedia, India) according to the Clinical and Laboratory Standards Institute (CLSI) recommendation for meropenem, amoxicillin, ceftazidime, piperacillin/tazobactam, gentamicin, tobramycin, amikacin, ciprofloxacin, and levofloxacin [18]. Also, MDR isolates were identified (MDR is defined by resistance to three or more antimicrobial classes) [18].

### 2.3. Biofilm Formation

#### 2.3.1. Phenotypic Evaluation

The microtiter plate (also called 96*-*well plate) assay for studying biofilm formation was performed. First, *P. aeruginosa* isolates were inoculated in 5 ml trypticase soy broth (TSB) (Gibco, USA) and incubated at 37°C for 24 h. Overnight cultures were diluted in TSB in order to get turbidity equal of 0.5 McFarland standard. 100 *μ*L of these dilutions was inoculated in 96 well microplates (JET BIOFIL, China). Sterile TSB and *P. aeruginosa* ATCC 27853 were used as negative and positive control. After incubation at 37°C for 24 h, the supernatant was removed, and wells were washed three times with normal saline solution (0.90% *w*/*v* of NaCl). Biofilm was fixed by using 96% ethanol and stained with crystal violet (1.5% *w*/*v*) for 20 minutes. The unbound stain was washed with water. The dye was solved in 150 *μ*L of 33% (*v*/*v*) acetic acid. By using a microplate reader, the optical densities (OD) of the wells (Anthos Labtec instruments, type: 22550) were determined in setting to 600 nm [19]. All assays were conducted in three series and repeated three times for each strain. Three standard deviations over the mean absorbance of negative control were considered as cut-off OD (OD_C_). Biofilm formation was categorized by the following formulas: if OD < ODc, the biofilm was not formed (negative), if ODc < OD < 2xODc, the biofilm was weak, if 2xODc < OD < 4xODc, the biofilm was moderate. If 4xODc < OD, the biofilm was strong [20].

#### 2.3.2. Screening for Biofilm-Related Genes

Bacterial DNA was extracted by boiling method [21]. The polymerase chain reaction (PCR) was performed to detect the presence of the genes encoding biofilm (*algD*, *psl-D*, *pel-F*, *Ppgl*, and *PAPI-1*), using primers listed in Table 1. Each 25 *μ*L reaction contains 2 *μ*L of DNA (10 *μ*g/mL), 10 *μ*L of Taq 2 × Master Mix (Amplicon, Denmark), 1 *μ*L of each forward and reverse primer with the concentration of 10 pmol/*μ*L, and 11 *μ*L of distilled water. The conditions for PCR reaction were initial denaturation at 94°C for 5 min, followed by 35 cycles at 94°C for 30 s, primer annealing at 56°C for *pslD*, 58°C for *algD*, *pelF*, *Ppgl*, and 59°C for *PAPI-1* and extension at 72°C for 45 s, and a final extension at 72°C for 7 min [20–22] The amplification products were analyzed with UV light after running for 45 minutes at 120 V on a 1% agarose gel [20].

### 2.4. Rep-PCR Fingerprinting Technique

The primers used for the Rep-PCR reaction were REP1R-I (5′-IIIICGICGICATCIGGC-3′) and REP2-I (5′-ICGICTTATCIGGCCTAC-3′) [23]. These primers have the nucleotide inosine at ambiguous positions in the REP consensus sequence. Inosine contains the purine base hypoxanthine and can base pair with A, C, G, or T. Oligonucleotides were designed by the Department of Pathology, University of Leeds, Leeds, United Kingdom. PCR condition was 3 min at 95°C; 30 cycles of 45 s at 94°C, 30 s at 50°C, and 45 s at 72°C; and finally, 5 min at 72°C. The PCR products were revealed by electrophoresis on a 1.5% agarose gel with 0.5x TBE at 3 hours with 60 voltage [17].

### 2.5. Statistical Analysis

Statistical analysis was performed by SPSS Statistics (Version 16). Chi-square or Fisher's exact test was used to determine any statistical association. Statistical significance was regarded as *p* values < 0.05. Also, Rep-PCR patterns were analyzed using GelJ software version 2.0 [24]. Isolates were assessed using UPGMA analysis and Dice coefficient; and finally, the relevant dendrogram was drawn. Isolates with a similarity coefficient equal to or above 70% were clustered as the same genotypes.

## 3. Results

In our study, 83 isolates (74.1%) from hospitalized patients and 29 isolates (25.9%) from outpatients were collected. The results of biofilm formation showed that 84.3% (70/83) of the strains isolated from hospitalized patients and 51.7% (15/29) of the strains isolated from outpatients were able to form biofilm (*p* value = 0.0004).

The biofilm formation assay among all isolates demonstrated that 85 strains (75.9%) were biofilm producers. In biofilm-producing isolates, 42.3% produced weak biofilms, 15.4% produced medium biofilms, and 42.3% formed strong biofilms. Also, 27 strains (24.1%) were nonproducers.

Antibiotic susceptibility test was performed only on strains isolated from hospitalized patients. Among *P. aeruginosa* isolates obtained from hospitalized patients, 45.8% (38/83) had MDR. MDR isolates among biofilm-producing strains (48.6%) were higher than nonforming strains (23%) but this difference was not statistically significant (*p* value = 0.089). Antibiotic susceptibility pattern in biofilm-positive and biofilm-negative isolates showed a high rate of antibiotic resistance to amoxicillin with 95.7% and 92.3%, respectively. The lowest antibiotic resistance rates in biofilm-positive and biofilm-negative isolates were seen against piperacillin/tazobactam (34.3%) and piperacillin/tazobactam and meropenem (15.4%), respectively. A significant association between the biofilm formation and resistance to ceftazidime and meropenem was shown in this study (*p* value = 0.048 and 0.033, respectively). Also, we investigated the antibiotic susceptibility pattern among isolates based on the intensity of biofilm formation. According to this, a significant association between strong biofilm formation and resistance to gentamicin and tobramycin was observed (*p* value = 0.023 and 0.047, respectively).

Based on PCR amplification results, *algD* gene was present in 78.6% (88/112) *P. aeruginosa* isolates, 87% (74/85) biofilm producer isolates, and 51.8% (14/27) nonproducers. Also, the occurrence of the *pelF* gene was 70.5% (79/112) among all isolates, 80% (68/85) among biofilm-producing isolates, and 40.7% (11/27) among nonbiofilm-producing isolates. In our study, 36.6% (41/112) of total isolates, 44.7% (38/85) of biofilm-positive isolates, and 11.1% (3/27) of biofilm-negative isolates carried the *pslD* gene. The gene encoding *Ppgl* was not detected in any of the isolates*. PAPI-1* gene was present in 77.6% (87/112) *P. aeruginosa* isolates, 85.9% (73/85) biofilm producer isolates, and 51.8% (14/27) nonproducer isolates. Finally, all three genes *algD*, *pelF*, and *pslD* were present simultaneously in 25.9% (29/112) isolates, 33% (28/85) biofilm-producing isolates, and 3.7% (1/27) nonbiofilm-producing isolates. Based on statistical analysis, a significant association between the presence of studied genes and biofilm formation was observed.

Dendrogram and gel electrophoresis images of Rep-PCR products from *P. aeruginosa* strains were shown in Figure 1. Rep-PCR fingerprints of 112 isolates generated 3 to 10 bands, and the molecular size ranged from 100 bp to more than 1 kb. Rep-PCR typing demonstrated that 112 *P. aeruginosa* isolates were classified into 57 types according to 70% cut-off. The predominant type was A which contained 15 isolates. Moreover, 7 isolates were clustered in genotype B, followed by C type (six), D (four), E (four), F (four), G (four), H (three), I (three), J (three isolates), and other genotypes were shown in Figure 1. Also, 35 isolates were distributed in scattered patterns and showed single types. The strains that were isolated from the Zanjan indicated the most diversity (27 types), followed by Sanandaj (26 types), Hamadan (13 types), Zahedan (9 types), and Mashhad city (8 types).

## 4. Discussion

*P. aeruginosa* is one of the most important pathogens causing serious infections in burn patients and the increase of MDR strains of *P. aeruginosa* in hospitals, especially the burn units are a major concern in controlling its infections [5]. Biofilm formation encourages the antibiotic resistance, partially due to the protective effect of a complex structure enclosing bacterial cells in an extracellular polymeric matrix, low cellular metabolic activity in biofilm structure, and the activity of efflux pumps that actively remove antimicrobial agents from the bacterial cells [25]. In *P. aeruginosa*, the biofilm matrix is comprised of *algD*, *pel*, and *psl* genes [9]. In the present study, the frequency of these genes and their association with biofilm formation were studied.

In this study, a significant relationship was observed between patients' hospitalization and biofilm formation (*p* value = 0.0004). Also, in our study, 75.9% of all isolates (85/112) were biofilm producers and 42.3% (36/112) of them were produced weak biofilms, 15.4% (13/112) produced medium biofilms, and 42.3% (36/112) formed strong biofilms. Also, 24.1% (27/112) of strains were nonproducers. Vasiljevic et al. investigated 163 *P. aeruginosa* strains for biofilm formation, of which 97.55% were biofilm-producer strains [26]. Among biofilm producers, 39.26% produced strong biofilms, 34.36% produced moderate biofilms, while 23.93% produced weak biofilms. Only 2.45% of studied strains were not biofilm producers [26]. In another study performed by Banar et al., 55 isolates (96.5%) of 57 *P. aeruginosa* isolates were biofilm producers, which indicated a higher rate than this study [20]. Also, Banar et al. reported that 30.9% of biofilm-producer isolates produced strong biofilms, 47.3% produced medium biofilms, and 21.8% of formed weak biofilms. Only 2 strains (3.5%) were nonproducers [20]. In a study carried out by Jabalameli et al., biofilm formation was detected in more than 96% of the strains among which 47% were strong biofilm producers, 26% were moderate, and 22.9% were weak biofilm producers [19]. In a study conducted by Corehtash et al., biofilm formation was seen in 92.4% of the *P. aeruginosa* isolates [27]. Also, the results of biofilm formation in the study performed by Delissalde and Amábile-Cuevas showed that after incubation for 8 and 24 hours, 14% (23 isolates) and 8% (13 isolates) of the isolates formed biofilm, respectively [28]. The discrepancy in the number of biofilm-producer strains and intensity of its formation may be related to differences in geographical areas, origin of infection, and sample size or the method of biofilm assay. In the present study, antibiotic susceptibility pattern in biofilm-positive and biofilm-negative isolates obtained from hospitalized patients showed a high rate of antibiotic resistance to amoxicillin with 95.7% and 92.3%, respectively. Similarly, Namuq et al. reported the highest antibiotic resistance to amoxicillin (98%) among *P. aeruginosa* isolates in their study [29]. The lowest antibiotic resistance rates in biofilm-positive and biofilm-negative isolates were seen against piperacillin/tazobactam (34.3 and 15.4%, respectively). This result agrees with Namuq et al. [29] who reported piperacillin/tazobactam resistance (5%), Hoque et al. [30] who reported (3.37%), and Direkel et al. [31] who reported (7%). Also, in a study performed by Delissalde and Amábile-Cuevas, the resistance of biofilm-producing strains against piperacillin/tazobactam was 35%, which was very similar to our results [28]. On the other hand, in the studies conducted by Jabalameli et al. and Corehtash et al., the resistance to piperacillin/tazobactam was reported to be 91.6% and 85.4%, respectively, which shows a higher rate than our results [19, 27]. The discrepancies in the level of antimicrobial resistance in different studies are probably related to the differences in the uncontrolled use of antibiotic in different regions and dissemination of drug resistance genes. Hence, before prescribing antibiotics, it is better to first check the status of antibiotic resistance in each geographical area and then selected the appropriate treatment. In the present study, the resistance to ceftazidime and meropenem in biofilm-producing strains was significantly higher than nonproducing strains. Similar to our results in Abdelraheem et al.'s study, the resistance to ceftazidime in biofilm-producing isolates was higher than nonforming isolates, but contrary to our results, no significant correlation was observed [32]. In our study, although the number of MDR isolates in biofilm-producing isolates was higher than nonforming isolates, no statistically significant association was observed between biofilm formation and MDR, while in studies performed by Corehtash et al. and Namuq et al., this association was seen as significant [27, 29]. In this study, based on PCR amplification results, *algD*, *pelF*, and *pslD* genes were present in 78.6%, 70.5%, and 36.6% of *P. aeruginosa* isolates. In a study carried out by Banar et al. [20], the frequency of these genes among 57 *P. aeruginosa* strains was as follows: *algD* (100%), *pelF* (93%), and *pslD* (54.6%). Also, in other studies conducted by Namuq et al., Ghadaksaz et al., and Zaranza et al, the frequency of the *algD* gene has been reported as 98%, 87.5%, and 39%, respectively [29, 33, 34]. Bacterial strains that carry the genes encoding the biofilm formation have the potential to cause severe infections. As a result, controlling these isolates is difficult and time-consuming. Circulating these isolates in population is a threat to public health.

There is no prevalence rate of *pslD* and *pelF* genes in other regions, but studies show that *pel* gene clusters are conserved among *P. aeruginosa* isolates [35], although, *psl* genes are not present in all isolates, which is somewhat in agreement with our results. The differences in reports of the distribution of these genes may be due to the different prevalent clones in each area, the geographical distribution. In our study, none of the isolates harbored *Ppgl*, and so far no study has reported the prevalence of this gene as one of the possible important factors in biofilm formation. Therefore, we suggest that this factor should be further investigated in future studies. In the current study, *PAPI-1* gene was present in 77.6% (87/112) of *P. aeruginosa* isolates. In a study conducted in Mexico, the frequency of *PAPI-1* gene was reported to be 81%, which is close to our results [36]. In two studies performed in Iran, the *PAPI-1* gene was detected in 35% and 14% of the isolates, which is not consistent with our results [37, 38]. This difference is probably due to differences in the type of *P. aeruginosa* infections in patients. Eventually, the frequency of all genes examined in biofilm-producer strains was higher than nonproducer strains, also a significant association was observed between the presence of these genes and biofilm formation (*p* < 0.001).

However, this genotypic technique allows the detection of gene-harboring strains independent of their expression. Accordingly, a positive result in the PCR only indicates the presence of the target gene, and may a strain has a target gene but that gene is not expressed [39]. So, it is better to determine more accurately the relationship between genes involved in biofilm and biofilm formation using real-time PCR, which is a quantitative technique that shows the amount of gene expression.

In our study, we performed Rep-PCR for the molecular typing of *P. aeruginosa* strains. It is a low-cost and rapid method that has proven as a valuable genotyping method for nonfermenting Gram-negative bacilli [40]. Analysis of Rep-PCR patterns indicated that the evaluated isolates were heterogeneous, relatively. Perhaps one of the reasons for the observation of such results is the ability of various strains of *P. aeruginosa* to survive in the hospital setting for a long time. Isolates obtained from Zanjan and Sanandaj were typed together in 7 clusters, which shows the most similarity between the five cities and may be due to the geographical proximity of the two cities and the spread of similar strains between the two cities.

The main limitation of our study is the lack of using a quantitative molecular technique such as real-time PCR to determine the expression of the studied genes. Because, PCR only indicates the presence of the gene, and may a strain has a gene but that gene is not expressed. However, reporting the percentage of biofilm-forming strains and their antibiotic resistance on the one hand and determining the frequency of genes involved in biofilm formation, on the other hand, can partially determine the status of strains in hospitals and improve the control and treatment of biofilm-forming and drug-resistant strains.

## 5. Conclusion

In this study, a high prevalence of biofilm producer isolates, implicated in hospitalized patients, is a serious problem that makes the treatment of *P. aeruginosa* infections difficult and complicated. Also, biofilm formation is highly associated with resistance to some antibiotics such as ceftazidime and meropenem. The *algD*, *pslD*, *pelF*, and *PAPI-1* genes have a significant role in biofilm formation, and in our study, a significant association between the presence of these genes and biofilm formation was observed. High diversity was observed in isolates with Rep-PCR.

## Figures and Tables

**Figure 1:** REP-PCR profiles of 112 *P. aeruginosa* isolates.

**Table 1:** Primers used for the PCR of the genes coding for biofilm among *P. aeruginosa* isolates.

Gene	Primer sequence (5′ to 3′)	Size of amplicon	Reference
*algD*	F-CTACATCGAGACCGTCTGCC	593	[20]
	R-GCATCAACGAACCGAGCATC		

*pelF*	F-GAGGTCAGCTACATCCGTCG	789	[20]
	R-TCATGCAATCTCCGTGGCTT		

*pslD*	F-TGTACACCGTGCTCAACGAC	369	[20]
	R-CTTCCGGCCCGATCTTCATC		

*Ppgl*	F-GTGGTGGGGACCTATACCGAA	327	This study
	R-GTAGTTGGCGACGAACAGGTA		

*PAPI-1*	F-CATCAACCGGATCGACGAAGT	462	This study
	R-GTCAACCCTCTGATCCAAAAAGTT		

## Data Availability

The data that support the findings of this study are available from the corresponding author upon reasonable request.
